RETRACTED

# Stretching Training Rehabilitation Has Potential to Alleviate Ankylosing Spondylitis in Mice by Inactivating the Wnt/*β*-Catenin Pathway

**DOI:** 10.1155/2022/3932504

**Published:** 2022-10-07

**Authors:** Yu Xie, Xiang Li, Qiuchi Zhang, Feng Guo, Yue Wang

**Affiliations:** ^1^Affiliated Hospital of Nanjing University of Chinese Medicine (Rheumatology Department, Jiangsu Province Hospital of Chinese Medicine), Nanjing 210029, China; ^2^Nanjing University of Chinese Medicine, Nanjing 210046, China; ^3^Affiliated Hospital of Nanjing University of Chinese Medicine (Neurology Department, Jiangsu Province Hospital of Chinese Medicine), Nanjing 210029, China

## Abstract

Ankylosing spondylitis (AS) is a chronic inflammatory disease characterized by invasion of the joints of the central axis that involves soft tissues and joints surrounding the spine. Stretching training rehabilitation (STR) has been widely applied for the treatment of AS. The Wnt/*β*-catenin signalling pathway is closely related to AS. In this study, we aimed to explore the potential molecular mechanisms underlying the protective effect of STR on AS both *in vitro* and *in vivo*. Male DBA/1 mice were employed to establish an AS animal model. Hematoxylin-eosin staining showed that STR reversed pathological damages in bone tissues and the total antioxidant capacity of AS mice and increased the antioxidant capacity by upregulating superoxide dismutase and malondialdehyde expression in DBA/1 mice. The MTT, RT-qPCR, and Western blotting results further indicated that STR improved the survival rate of cells by downregulating the expression of target genes in the Wnt/*β*-catenin pathway and by inhibiting cell inflammation and apoptosis. In conclusion, our findings indicated that STR treatment might be an effective therapeutical strategy for AS.

## 1. Introduction

Ankylosing spondylitis (AS) is a prototypical disease of spinal arthritis (SpA) [1]. It is a chronic inflammatory disease characterized by invasion of the joints of the central axis that involves soft tissues and joints surrounding the spine [2, 3]. The main clinical manifestations are trunk pain and joint swelling and pain at the early stage of the disease, and the main manifestations of the disease are stiffness of the spine and joints [4]. Currently, the pathogenic mechanism for AS is not completely clear. Moreover, an effective cure is unavailable, which has a serious effect on patients' health and daily life, and thus, it is called “undead cancer” [5]. The main goal of AS treatment is to control inflammation as early as possible to improve function and reduce deformity. Various ligaments of the human body will be opened during the stretching process, heating and sweating will occur through physical activity, and then, the whole body will be adjusted to the best state, which is convenient for larger and more intense exercises [6, 7]. Stretching is a common method used in flexibility training. Through good stretching, the joints and muscles of the body will become more flexible, which may effectively improve the stiffness of the limbs and improve the flexibility of the body [8, 9]. A radical cure has not been developed for AS. Appropriate intervention measures are used to control symptoms, restore and maintain physiological functions, delay disease progression, reduce the disability rate, and improve quality of life which are the main goals of treatment and care [10]. Studies conducted abroad have confirmed that stretching training improves the physical activity of patients, delays spinal sclerosis, and promotes disease recovery [11]. This study observes the therapeutic effect of stretching exercise prescriptions on patients with AS and the specific mechanism of disease treatment.

RETRACTED

Recent studies have shown that the Wnt/*β*-catenin signalling pathway is closely related to AS [12]. Wnt/*β*-catenin proteins bind to receptors located on the cell membrane and activate intracellular signalling pathways through autocrine or paracrine mechanisms, resulting in modulation of the expression of target genes [13]. The Wnt/*β*-catenin signalling pathway has been conformed to regulate cell proliferation, differentiation, inflammation, and apoptosis in different human diseases and cancers [14].

In this study, DBA/1 mice were used to experimentally verify the regulatory effect of stretching exercise on Wnt/*β*-catenin activity, inflammation, and cell apoptosis. We found that stretching exercise improved the antioxidant capacity of AS mice. We extracted synovial cells from the ankle joint of mice and added pathway inhibitors and agonists to explore the effect of stretching exercise on Wnt/*β*-catenin activity and cell proliferation. Our results indicated that stretching exercise might be an effective therapeutical strategy for AS.

## 2. Materials and Methods

### 2.1. Animals and Groups

Fifty male DBA/1 mice (Vital River, Beijing, China) of SPF grade aged 26 weeks, with an average body weight of 21.7 ± 1.4 g, were used. The culture room temperature was set to 22–25°C with a humidity of 50-70%, and animals were provided free access to food and drinking water. Fifty DBA/1 mice were randomly divided into five groups with 10 mice in each group: (1) the normal mouse group (normal group), (2) the unprocessed AS model mouse group (model group), (3) AS model mice receiving routine nursing care+pressure-relief stretch (positive control group), (4) AS model mice treated with routine nursing care+pressure-relief stretch+simulated stretching training (stretching exercise group), and (5) normal mice undergoing stretching exercise. The model group and the normal group were raised normally every day [15]. Stretching exercise was performed as described. The mouse was gently stretched in the direction of the lower limbs to fully stretch the mouse. Two sessions were performed per day, and each session included 10 stretches in 5 d/week for 12 weeks. In addition, the pressure-relief stretch was largely mimicking the actions of the stretching exercise procedure. However, the mouse was never stretched in the direction of the lower limbs in order to avoid any pressures induced by the stretching motion.

RETRACTED

### 2.2. Hematoxylin-Eosin (HE) Staining

Mice were anaesthetized and then sacrificed by dislocation of the cervical vertebra. Ten minutes after confirming the death of mice, the heart of each mouse was sequentially cardiac perfused with 10 mL each of 1x PBS and 4% paraformaldehyde via the vena cava. Then, the bone tissue was removed and placed in a 30% sucrose solution overnight. After the tissue sunk to the bottom, it was embedded at -80°C. Continuous coronal sections were cut using a freezing slicer (Thermo Fisher Scientific, Waltham, MA, USA). Sections were fixed with 70%, 80%, and 90% alcohol for 5 s, stained with hematoxylin for 15 s, incubated with 1% hydrochloric acid alcohol for 5 s and 0.5% ammonia for 10 s, and stained with eosin for 5 s. Next, sections were washed with 1x PBS, dehydrated with 70%, 80%, and 90% alcohol for 5 s, and sealed with neutral gum. The final stained sections were observed under a microscope (Nikon, Tokyo, Japan) [16].

### 2.3. Total Antioxidant Status (TAS) Determination

Serum samples were prepared using a standard venous blood sampling protocol. Blood in mice was collected through the tail vein (0.1 mL/mouse) after anaesthesia. After centrifugation at 3,000 × g for 10 min at 4°C, the serum was obtained then transferred to a clean tube, followed by storage at −80°C until use. The FRAP chemical colorimetry assay was chosen. The serum samples were analysed using the total antioxidant status (TAS) test kit (Sigma-Aldrich, Saint Louis, MO, USA) for the TAS determination. The operation steps are described below: (1) Preparation: place the required specimens and reagents at room temperature (18-25°C) and allow them to slowly rewarm. (2) The test wavelength of the automatic biochemical analyser (HITACHI 7600-210) was set to 580-605 nm. (3) A blank control was prepared. After calibration (2.18 mmol/L) and quality control (1.47 mmol/L), the quality control range (*x* ± *s*) was 1.46 ± 0.14 mmol/L, and the quality control result was 1.41 mmol/L. Thus, both calibration and quality control were appropriate for the assay. (4) Serum samples from each group of mice were loaded into the sample rack, and their TAS levels were measured [17, 18].

RETRACTED

### 2.4. Superoxide Dismutase (SOD) Assay

Serum samples were prepared using a standard venous blood sampling protocol. Blood in mice was collected through the tail vein (0.1 mL/mouse) after anaesthesia. After centrifugation at 3,000 × g for 10 min at 4°C, the serum was obtained then transferred to a clean tube, followed by storage at −80°C until use. In an alkaline environment, pyrogallol produces its own oxidation color reaction. The intensity of the color reaction caused by self-oxidation is high or low, depending on the concentration of superoxide anion radicals released during the reaction. Therefore, a high concentration of superoxide anion radicals is released during the reaction, and vice versa, a low concentration of superoxide anion radicals. Briefly, 4.5 mL of Tris-HCl-EDTA buffer, pH 8.2, was placed in a 10 mL colorimetric tube, incubated at 25°C for 10 min, and then added to 10 mL of a 45 mmol/L pyrogallol solution at 25°C. The optical density value was measured at a wavelength of 325 nm once every 30 s for a total of 4 min to obtain the autooxidation rate of pyrogallol in OD_A_/min. At the same time, a blank test was performed with 10 mmol/L hydrochloric acid. For this analysis, 4.5 mL of the Tris-HCl-EDTA buffer solution, pH 8.2, was placed in a 10 mL colorimetric tube and incubated at 25°C for 10 min. Ten milliliters of sample solution at 25°C was mixed quickly with the buffer, and the density value was measured at a 325 nm wavelength at 30 s and 4 min. The rate of change in the optical density value was reported as OD_B_/min. SOD activity (U/mL) = [(OD_A_‐OD_B_)/OD_A_] × 100% ÷ 50% × *V*_1_ ÷ *V*_2_ × *n*. Here, *V*_1_ is the total volume of the reaction solution (mL), *V*_2_ is the measured sample volume (mL), *n* is the sample diluent multiple, OD_A_ is the autooxidation rate of pyrogallol, and OD_B_ is the change rate of the sample optical density value [19].

### 2.5. Malondialdehyde (MDA) Assay

Serum samples were prepared using a standard venous blood sampling protocol. Blood in mice was collected through the tail vein (0.1 mL/mouse) after anaesthesia. After centrifugation at 3,000 × g for 10 min at 4°C, the serum was obtained then transferred to a clean tube, followed by storage at −80°C until use. Malondialdehyde (MDA) was heated with thiobarbituric acid (TBA) under acidic conditions (100°C, 20-60 min) to produce pink substances, and the maximum absorption peak at 535 nm was recorded to calculate the amount of lipid peroxidation. Briefly, 0.4 mL of the test solution was added to 3.6 mL of lecithin solution; then, 0.4 mL of FeSO_4_ solution was added to catalyse the oxidation reaction, mixed, and placed in a constant temperature water bath shaker at 37°C in the dark for 1 h, followed by the addition of 1 mL of trichloroacetic acid solution. Next, 1 mL of TBA was added, shaken well, boiled in a water bath for 15 min, cooled quickly, and centrifuged at 5000 r/min for 10 min, and the supernatant was collected, and the absorbance Ax was measured at 535 nm. The blank tube contained distilled water instead of the sample to be tested, the operation method was the same as that of quality control, and the absorbance A0 of the blank tube was measured. Three parallel measurements were performed [19].

RETRACTED

### 2.6. Synovial Tissue Extraction and Cell Culture

Synovial tissues were minced from mice in four different groups (normal, normal+stretching exercise, model, and model+stretching exercise) with ophthalmic scissors, digested with type I collagenase (1 mg/mL), and digested in a 37°C, 5% CO_2_ cell incubator for 2 to 4 h. The sample was filtered using a 100 *μ*m pore size filter and a large and small cell strainer and then centrifuged to pellet the cells. DMEM (Invitrogen, Carlsbad, CA, USA) containing 10% FBS (Invitrogen) was used to resuspend the cells and transferred to a cell culture flask for culture; the medium was changed every 2 to 4 days. The cell morphology and growth of the primary and postpassage cells were observed. When the cells reached passages 3-4, they were digested to prepare a single cell suspension with a density of 1 × 10^5^ cells/mL. Additionally, LiCl (10 mmol/L; Sigma-Aldrich) or IWR (10 mmol/L; Sigma-Aldrich) was added to cells of the model or model+stretching exercise groups [20].

### 2.7. 3-(4,5)-Dimethylthiahiazo(-z-y1)-3,5-di-phenytetrazoliumromide (MTT) Assay

Three replicate wells in each group were prepared; 100 *μ*L of medium was added to each well and incubated overnight. The MTT reagent (Beyotime, Shanghai, China) was added to each well and incubated for 4 h in the dark; the culture solution was discarded, DMSO solution was added and shaken for 10 min, and finally, the absorbance was measured at 570 nm using a microplate reader (Molecular Devices, USA) [21]. All experiments were performed in biological triplicates, and data are representative of three independent experiments.

### 2.8. RT-qPCR Analysis

Total RNA was isolated from bone tissues and synovial cells of mice in each group using the TRIzol reagent (Invitrogen) and converted cDNAs using the OneScript Reverse Transcriptase OneScript cDNA Synthesis Kit (Abcam, Cambridge, MA, USA). Twenty-five microliters of Dream Taq PCR Master Mix (Abcam), 1.5 *μ*L of forward and reverse primers (Ribobio, Guangzhou, China), 2 *μ*L of cDNAs, and 20 *μ*L of nuclease-free water were included in the amplification reaction mixture (50 *μ*L), and the PCR conditions were as follows: 95°C (2 min, one cycle); 35 cycles of 95°C (30 s), 58°C (30 s), and 72°C (1 min) (21) [15]; and a final cycle of 72°C (10 min). The mouse *β*-actin gene was used as an internal control. The following primer sequences were used: *β*-catenin, F: 5′-CCACTCCAGGAATGAAGG-3′, R: 5′-AGCAGTCTCATTCCAAGC-3′; TNF-*α*, F: 5′-ATAAGAGCAAGGCAGTGGAG-3′, R: 5′-TCCAGCAGACTCAATACACA-3′; IL-17, F: 5′-AGCCAGAGTCCTTCAGAGAG-3′, R: 5′-TCCTTAGCCACTCCTTCTGT-3′; Bcl-2, F: 5′-CTGGTGGACAACATCGC-3′, R: 5′-GGAG-AAATCAAACAGAGGC-3′; and *β*-actin, F: 5′-TCACCATCTTCCAGGAGCGAG-3′, R: 5′-TGTCGCTGTTGAAGTCAGAG-3′. All experiments were performed in biological triplicates (*n* = 6), and data are representative of three independent experiments. The relative transcript abundances (2^−*ΔΔ*CT^) were calculated based on the equation 2^−∆CT^ (∆CT = CT_target gene_–CT_*β*‐actin_). The differences were determined using unpaired Student's *t*-test for comparisons between different groups. A *P* value of <0.05 was regarded as statistically significant.

RETRACTED

### 2.9. Western Blot Assay

Western blotting was used to detect the relative protein expression. After extracting the total protein from the bone tissue, 10-25 *μ*L was added to each well for sodium dodecyl sulphate-polyacrylamide gel electrophoresis (SDS-PAGE) (60 V, when the distance migrated by bromophenol blue was approximately 1 cm from the bottom of the separation gel, stop electrophoresis) followed by wet transfer to polyvinylidene fluoride (PVDF) membranes (Millipore, Billerica, MA, USA) at 120 mA (2-3 h). The membrane was blocked with a solution containing 5% skim milk powder at room temperature for 1 h and rinsed with TBST 3 times. The membrane was incubated with antibodies against *β*-catenin (Abcam, ab32572, 1 : 5000), TNF-*α* (Abcam, ab183218, 1 : 1000), IL-17 (Abcam, ab79056, 1 : 2000), and *β*-actin (Abcam, ab8227, 1 : 1000) at 4°C overnight, rinsed with TBST 3 times, incubated with the secondary antibody (Abcam, ab6721, 1 : 2000) in the dark at room temperature for 2 h, and rinsed with TBST 3 times in the dark. Bands were visualized with electrochemiluminescence (ECL) (Pierce, Rockford, IL, USA), and analysed by ImageJ (v1.8.0; National Institutes of Health) [22, 23].

### 2.10. Statistical Analysis

Statistical analyses were performed using GraphPad Prism software (version 7.0). Data are presented as the means ± SD (standard deviations). Differences and comparisons between multiple groups were analysed using one-way ANOVA followed by a post hoc test (Tukey's test). *P* < 0.05 indicated a significant difference.

RETRACTED

## 3. Results

### 3.1. Stretching Exercise Reverses the Pathological Damage to Bone Tissues in AS Mice

The Achilles tendon showed no infiltration of inflammatory cells and fibroblasts and a normal morphological structure in the normal group. The model group presented varying degrees of cartilage and bone formation, inflammatory cells, and fibroblast-like infiltration of attachment points. The mice in the stretching exercise group had small Achilles tendon tissues that more frequently contained scattered infiltrating lymphocytes, and cartilage and bone formation were rare (Figures 1(a) and 1(b)). Therefore, the therapeutic effect on the stretching exercise group was better than that on the normal group. These results indicate that stretching exercise reverses pathological injuries in an AS mouse model.

### 3.2. Stretching Exercise Increases the Antioxidant TAS of AS Mice by Upregulating SOD Expression and Inhibiting MDA Expression

We examined the antioxidant effect of stretching exercise on mice with AS and found a significantly lower serum level of the antioxidant TAS in model mice than in normal mice, while mice in the stretching exercise group had significantly increased TAS levels (Figure 1(c)). Based on these results, stretching exercise improves the antioxidant capacity of AS mice. We further measured the serum SOD and MDA levels in each group of mice to verify the effect of stretching exercise on the antioxidant capacity of AS mice. The serum level of the antioxidant SOD was significantly decreased in the model group when compared with the normal mice (Figure 1(d)). However, after stretching exercise treatment, AS mice exhibited a significant increase in SOD levels compared with the model group (Figure 1(d)). The MDA levels were also determined in mice of each group. Serum levels of the MDA in mice from the model group were significantly higher than those in healthy subjects (Figure 1(e)). However, stretching exercise treatment significantly decreased MDA levels in AS model mice (Figure 1(e)).

### 3.3. Stretching Exercise Downregulates the Wnt/*β*-Catenin Signalling Pathway in AS Mice and Inhibits the Expression of Inflammatory Factors

Total RNA and proteins were extracted from mouse plasma samples, and the relative mRNA expression levels of inflammation-related factors were detected using RT-qPCR. As shown in Figure 2(a), compared with the normal group, the expression levels of TNF-*α* and IL-17 in the model group were increased significantly and were then significantly reduced after stretching exercise. Meanwhile, the expression level of the *β*-catenin mRNA in the model group was significantly higher than that in the control group, while *β*-catenin expression in the stretching exercise group was significantly decreased. The relative protein levels were detected using Western blot assays (Figure 2(b)). Compared with the normal control group, the levels of inflammation-related factors TNF-*α*, IL-17, and *β*-catenin were significantly elevated in the model group, while stretching exercise reduced their levels.

RETRACTED

### 3.4. Stretching Exercise Improves the Viability of Synovial Cells

We extracted synovial cells from the ankle joint tissues of mice from three groups (normal, model, and model+stretching exercise) and added LiCl (agonist of the canonical Wnt signalling) and IWR (inhibitor of the canonical Wnt signalling) to the cells of the model group and the model+stretching exercise group to study the mechanism underlying the therapeutic effect of stretching exercise on AS. MTT results showed that cell in the model group has lower viability than that in the normal group. LiCl decreased cell viability while IWR or stretching exercise increased cell viability. Stretching simulation reversed the effect of LiCl and aggravated the effect of IWR on cell viability (Figure 3).

### 3.5. Stretching Exercise Shows Anti-inflammatory Effect and Inhibits Cell Apoptosis by Blocking the Wnt/*β*-Catenin Signalling Pathway

We extracted synovial cells from the ankle joint tissues of mice from four groups (normal, normal+stretching exercise, model, and model+stretching exercise) and added LiCl and IWR to the cells of the model group and the model+stretching exercise group. The RT-qPCR results revealed that cells in the model group showed increased TNF-*α*, IL-17, and *β*-catenin mRNA expression. Stretching exercise decreased TNF-*α*, IL-17, and *β*-catenin mRNA levels in both normal synovial cells and model cells. LiCl increased TNF-*α*, IL-17, and *β*-catenin mRNA expression while IWR decreased TNF-*α*, IL-17, and *β*-catenin mRNA expression in model cells. Stretching exercise rescued the effects of LiCl and aggravated the effects of IWR on TNF-*α*, IL-17, and *β*-catenin mRNA expression in model cells (Figures 4(a)–4(c)).  Figure 4(d) revealed that cells in the model group showed decreased Bcl-2 mRNA expression. Stretching exercise increased Bcl-2 mRNA in both normal synovial cells and model cells. LiCl decreased Bcl-2 mRNA expression while IWR increased Bcl-2 mRNA expression in model cells. The stretching exercise rescued the effects of LiCl and aggravated the effects of IWR on Bcl-2 mRNA expression in model cells. Western blotting was further conducted to reveal the protein levels of TNF-*α*, IL-17, and *β*-catenin, and the results were the same as the RT-qPCR results (Figures 5(a)–5(d)). These results indicated that stretching training shows an anti-inflammatory effect and inhibits cell apoptosis by blocking the Wnt/*β*-catenin signalling pathway.

RETRACTED

## 4. Discussion

AS is a systemic disease that is mainly caused by chronic inflammation of the joints [24, 25]. Its incidence is mostly related to specific genetic factors, endocrine disorders, autoimmune function, and the external environment [26]. The cause of the disease has not been elucidated. Currently, clinicians generally believe that early and timely treatment and effective control of disease progression are particularly important for patients [26]. Stretching training is important for fitness exercises because it relieves fatigue symptoms, accelerates the rate of lactic acid decomposition in the body after exercise, and fully stretches muscle tissue [27, 28], along with reducing the incidence of sports injuries, preventing blood stasis, and ensuring the safety of sports while enhancing the body's ability in all aspects [29]. The body should not feel pain during stretching training [30]. Usually, when the body feels comfortable, a sufficient approach is to ensure that the muscles have a certain degree of tension. Studies have shown that stretching training exerts a good therapeutic effect on AS [31, 32].

In this paper, DBA/1 mice were used as a focus for follow-up research to verify the specific mechanism by which stretching training inhibits inflammation and apoptosis through the Wnt/*β*-catenin signalling pathway. AS is a type of rheumatism characterized by chronic inflammation of the axial joint and may involve the internal organs and other tissues [33]. TNF-*α*, IL-6, IL-8, and IL-17 have been identified to be overexpressed in AS patients [34]. Furthermore, in AS patients, neutrophils are activated so that reactive oxygen species are generated, resulting in oxidative stress [35]. Naringin represses AS progression via inhibiting inflammation and oxidative stress in mice [36]. We found that stretching training effectively improves the antioxidant capacity of AS mice and effectively alleviates inflammation associated with AS. It reduces the pathological damage of AS and downregulates TNF-*α*, IL-17, and *β*-catenin expression. The Wnt pathway has been confirmed to be closely associated with AS development [37]. For example, miR-148a-3p facilitates osteogenic differentiation of fibroblasts in AS by activating the Wnt pathway and targeting DKK1 [38]. miR-22-3p by M2 macrophage-derived extracellular vesicles facilitates the development of AS through the Wnt/*β*-catenin pathway [39]. We subsequently extracted synovial cells from DBA/1 mice and treated some cells with Wnt/*β*-catenin inhibitor or agonist. Compared with the model group, the expression of the TNF-*α*, IL-17, and *β*-catenin was increased by LiCl and decreased by IWR. Stretching exercise rescued the effects of LiCl and aggravated the effects of IWR on TNF-*α*, IL-17, and *β*-catenin expression. Expression of antiapoptotic factor Bcl-2 showed the opposite trend under the same treatment. These results indicated that the therapeutical effect of stretching exercise on AS is mediated by the Wnt/*β*-catenin axis. Stretching exercise inhibits cell inflammation and apoptosis through blocking the Wnt/*β*-catenin signalling pathway.

RETRACTED

Based on this study, stretching exercise could significantly improve the antioxidant capacity of AS mice by increasing the serum level of TAS, SOD, and MDA *in vivo*. This provides an interesting point worthy of discussion and further investigation. Many diseases, such as cardiovascular diseases, neurodegenerative disease, cancer, diabetes, atherosclerosis, inflammatory diseases, and premature aging, are all related to oxidative stress [40]. However, there is little information available on the potential indicators for the application of stretching exercise in the treatment of oxidative stress-related diseases, and few mechanisms have been excavated. Therefore, our results might enlighten the research and clinical treatment of oxidative stress-induced bone-related diseases and have a certain significance of reference for other oxidative stress-induced diseases.

In summary, we experimentally verified the regulatory effect of stretching exercise on Wnt/*β*-catenin signalling and its inhibition of inflammation and the occurrence of apoptosis. Stretching exercise improves the antioxidant capacity of AS mice by regulating Wnt/*β*-catenin signalling (Figure 6). Our results indicated that stretching exercise might be an effective therapeutical strategy for AS treatment, although further clinical evidence is needed.

## Figures and Tables

**Figure 1:** Effect of stretching exercise on pathological changes in the Achilles tendon of each group of AS mice. Forty DBA/1 mice were randomly divided into four groups (*n* = 10/group): the normal mouse group (namely, normal group), unprocessed AS model mouse group (namely, model group), AS model mice receiving routine nursing care+pressure-relief stretch used as a control group (namely, positive control group), and AS model mice treated with routine nursing care+pressure-relief stretch+simulated stretching training (namely, stretching exercise group). (a) Pathological observation of the Achilles tendon using H&E staining method to detect osteogenesis. Arrows (in black) indicate the locations of the infiltration of inflammatory cells, fibroblasts, and cartilage and bone formation. Bar: 100 *μ*m. (b) Cell infiltration in different groups was detected. (c–e) The effect of stretching exercise on the antioxidant capacity of AS mice. The serum TAS (c), SOD (d), and MDA (e) levels were determined and compared between different groups of DBA/1 mice. Data are representative of three independent experiments. Data are presented as means ± SD. Comparisons between multiple groups were analysed using one-way ANOVA followed by a post hoc test (Tukey's test). ^∗∗^*P* < 0.01 and ^∗∗∗^*P* < 0.001 vs. control; ^#^*P* < 0.05 and ^###^*P* < 0.001 vs. model.

RETRACTED

**Figure 2:** Stretching exercise downregulates the expression of *β*-catenin and inflammatory factors in AS mice. (a) TNF-*α*, *β*-catenin, and IL-17 mRNA expression levels were detected using RT-qPCR. (b) Protein expression levels were detected using Western blot assays. Mouse *β*-actin was used as an internal reference. Data are representative of three independent experiments. Data are presented as means ± SD. Differences and comparisons between multiple groups were analysed using one-way ANOVA followed by a post hoc test (Tukey's test). ^∗∗∗^*P* < 0.001 vs. control; ^###^*P* < 0.001 vs. model.

**Figure 3:** The effect of stretching exercise treatment on the survival rate of synovial cells was determined using the MTT assay. Synovial cells were extracted from the ankle joint tissues of mice (normal, model, and model+stretching exercise). Cells in the model and model+stretching exercise groups were treated with LiCl or IWR. All experiments were performed in triplicates, and data are representative of three independent experiments. Data are presented as means ± SD. Differences and comparisons between multiple groups were analysed using one-way ANOVA followed by a post hoc test (Tukey's test). ^∗∗∗^*P* < 0.001 vs. control; ^#^*P* < 0.05 and ^##^*P* < 0.01 vs. model; ^&&^*P* < 0.01 and ^&&&^*P* < 0.001 vs. model+stretching exercise.

**Figure 4:** Expression of target genes in the Wnt/*β*-catenin signalling pathway. Total RNA was extracted from synovial cells from mice in four groups (normal, normal+stretching exercise, model, and model+stretching exercise). Cells in the model and model+stretching exercise groups were treated with LiCl or IWR. (a) TNF-*α*, (b) IL-17, (c) *β*-catenin, and (d) Bcl-2 mRNA expression levels were determined using RT-qPCR. The *β*-actin mRNA was used as an internal reference. All experiments were performed in triplicates, and data are representative of three independent experiments. Data are presented as means ± SD. Differences and comparisons between multiple groups were analysed using one-way ANOVA followed by a post hoc test (Tukey's test). ^∗^*P* < 0.05, ^∗∗^*P* < 0.01, and ^∗∗∗^*P* < 0.001 vs. control; ^#^*P* < 0.05, ^##^*P* < 0.01, and ^###^*P* < 0.001 vs. model; ^&^*P* < 0.05, ^&&^*P* < 0.01, and ^&&&^*P* < 0.001 vs. model+stretching exercise.

RETRACTED

**Figure 5:** Western blot assay of the levels of target proteins involved in the Wnt/*β*-catenin signalling pathway: (a) TNF-*α*, IL-17, and *β*-catenin protein bands. (b) TNF-*α*, (c) IL-17, and (d) *β*-catenin quantified protein expression levels. The *β*-actin protein was used as an internal reference. Total protein was extracted from synovial cells from mice in four groups (normal, normal+stretching exercise, model, and model+stretching exercise). Cells in the model and model+stretching exercise groups were treated with LiCl or IWR. All experiments were performed in triplicates, and data are representative of three independent experiments. Data are presented as means ± SD. Differences and comparisons between multiple groups were analysed using one-way ANOVA followed by a post hoc test (Tukey's test). ^∗^*P* < 0.05, ^∗∗^*P* < 0.01, and ^∗∗∗^*P* < 0.001 vs. control; ^#^*P* < 0.05, ^##^*P* < 0.01, and ^###^*P* < 0.001 vs. model; ^&^*P* < 0.05 and ^&&^*P* < 0.01 vs. model+stretching exercise.

**Figure 6:** Summary of the cellular response and potential molecular mechanism of stretching training treatment on AS model. Stretching training treatment improved the viability of synovial cells *in vitro* and downregulated the expression of target genes in the Wnt/*β*-catenin signalling pathway, inhibited inflammation and cell apoptosis, and relieved pathological damages in bone tissue in DBA/1 mice of AS.

## Data Availability

Data analysed in the current study are available from the corresponding author on reasonable request.
